# Efficiency of *Coriandrum sativum* (Linn.) and *Petroselinum crispum* (Mill.) in Enhancing Iron Absorption: An *In Silico* and *In Vitro* Approach

**DOI:** 10.1155/2022/7359081

**Published:** 2022-04-30

**Authors:** T. Sangeetha, K. Syed Ibrahim, S. Deepa, B. Balamuralikrishnan, M. Arun, S. Velayuthaprabhu, K. M. Saradhadevi, A. Vijaya Anand

**Affiliations:** ^1^Department of Human Genetics and Molecular Biology, Bharathiar University, Coimbatore, Tamil Nadu, India; ^2^PG & Research Department of Botany, PSG College of Arts and Science, Coimbatore, Tamil Nadu, India; ^3^Department of Food Science and Biotechnology, Sejong University, Seoul, Republic of Korea; ^4^Department of Obstetrics and Gynaecology, Centre for Perinatal and Reproductive Medicine, University of Perugia, Perugia, Italy; ^5^Department of Biotechnology, Bharathiar University, Tamil Nadu, Coimbatore, India; ^6^Department of Biochemistry, Bharathiar University, Tamil Nadu, Coimbatore, India

## Abstract

*Coriandrum sativum* (Linn.) and *Petroselinum crispum* (Mill.) are the common herbs used for culinary purposes in daily life. The chlorophyll pigment in plants is being identified with various medicinal values, whereas iron is an essential micronutrient for the proper metabolism of the human body. The current research has been aimed at predicting the role of *C. sativum* and *P. crispum* in enhancing iron absorption *via* an *in vitro* approach. *C. sativum* and *P. crispum* have been analyzed for their capability of being a source of chlorophyll and iron concentration. The extracts prepared from solvents like carbinol, petroleum ether, and water were subjected to the identification of phytoconstituents through gas chromatography-mass spectrometry analysis, and the identified compounds were subjected to *in silico* studies against the iron-binding receptor, transferrin, to depict the binding affinity of the identified compounds. The carbinol extract was then put through *in vitro* analytical studies in Caco2 cell lines with a concentration of 500 µg/ml. Current research has shown that the leaves of *C. sativum* and *P. crispum* are an excellent source of chlorophyll and iron and has also suggested that these herbs efficiently enhance the absorption of iron in human intestinal cells.

## 1. Introduction

*Coriandrum sativum* (Linn.), commonly called coriander, and *Petroselinum crispum* (Mill.), commonly called Chinese coriander or parsley, belong to the Apiaceae family.  Table 1 shows the family characterization of *C. sativum* and *P. crispum.* These two plants are most efficiently used in the medicinal field as well as in the culinary areas [1]. The phytochemical compounds present in these plants are being identified to have various medicinal purposes, including anti-inflammatory, neuroprotectivity, antidiabetic, anticancer, antibacterial, and antifungal activities [2–5]. One of the most important micronutrients needed by the human body is iron [6]. Approximately about 8.7 mg and 14.8 mg of iron are needed per day by men and women, respectively [7]. The improper iron supplementation affects the transportation of oxygen directly since iron is an essential component in the formation of erythrocytes, which are composed of a protein called hemoglobin that is majorly involved in oxygen transport [8]. Deficiency in the iron content may be due to various reasons like improper iron absorption by the intestine, excess loss of iron, or improper intake of iron. The duodenum and jejunum are the parts of the small intestine involved in iron absorption [9]. Anemia is the predominant clinical condition caused as a result of iron deficiency, whereas iron deficiency may also be life-threatening in the event of occurring as a comorbidity along with heart and kidney failure [10]. The concentrations of iron in the herbs *C. sativum* and *P. crispum* are found to be present in significant concentrations, yet the clinical significance and pathophysiology of iron absorption in the intestines from these herbs are still unclear. Hence, the human colon adenocarcinoma (Caco2) cell lines, which are mainly derived from colon carcinoma, are mainly used in studies related to the intestinal epithelial barrier. The current study has been aimed at analyzing the effectiveness of the leaf extracts of *C. sativum* and *P. crispum* in the absorption of iron by human intestinal cells *via in vitro* studies using Caco2 cell lines. The iron absorption enhancement by using the plant extracts may provide an effective and easy way of treating the acquired iron deficiency in human individuals.

## 2. Materials and Methods

### 2.1. Plant Collection

The seeds of plants *C. sativum* and *P. crispum* have been sown and grown in partial sunlight, and the plant identification has been done after the plant has reached its complete growth (Plant Identification Number: 2998, 2999; Department of Botany, St. Joseph's College, Tiruchirapalli, Tamil Nadu, India). The leaves of the plants had been collected just before the flowering stage, and the fresh leaves were subjected to chlorophyll estimation, while the remaining leaves were dried in the shade for further analysis.

### 2.2. Chlorophyll Estimation

The fresh leaves of *C. sativum* and *P. crispum* were crushed into a fluid by using 80% acetone in a mortar and pestle. The fluid was then centrifuged and the supernatant was collected in a 100 ml standard flask. The centrifugation with 80% acetone has been repeated until a clear supernatant is obtained. The obtained supernatant was then made up to 100 ml with 80% acetone and the solution was taken for colorimetric analysis at 645 nm and 663 nm. The concentration of chlorophyll has been calculated using the Arnon formula [11], chlorophyll content = [20.2 (*A*_645_) + 8.02 (*A*_663_)/1000 x weight] *x* volume, with the obtained values.

### 2.3. Iron Estimation

The shade-dried leaves of *C. sativum* and *P. crispum* were used for the estimation of iron by using the thiocyanate method [12]. 1 in 10 dilutions of the stock standard, which was prepared by using ferrous ammonium sulphate and 30% sulfuric acid in demineralized water, was used as the working standard solution, followed by the addition of 30% sulfuric acid, potassium persulphate, and potassium thiocyanate as reagents during the analysis. The optical density values were recorded at 540 nm in the colorimeter.

### 2.4. Molecular Docking

The dried leaves of *C. sativum* and *P. crispum* were subjected to soxhlet extraction by using three different solvents, carbinol, petroleum ether, and water. The extracts obtained were then subjected to gas chromatography-mass spectrometry (GC-MS) analysis. The phytochemical compounds were then subjected to virtual screening using the SwissADME software to scrutinize the compounds based on pharmacokinetic properties and drug-likeness, which includes the Lipinski rule. The scrutinized compounds are then analyzed for their binding capacity with the iron-binding receptor, transferrin (1KAS), *via* molecular docking by using AutoDock Vina (version 1.1.2).

### 2.5. *In Vitro* Studies

The culturing of Caco2 cells was performed using Dulbecco's modified Eagle's medium with high glucose containing 10% fetal bovine serum. The cultured cells were then treated with 0.25% trypsin and centrifuged at 300g. Then 200 *μ*l of the suspension obtained was loaded in a 96-well microtiter plate and incubation at 37^o^C in 5% carbon dioxide for 24 hours was carried out. The five different test concentrations (62.5 *μ*l, 125 *μ*l, 250 *μ*l, 500 *μ*l, and 1000 *μ*l) of the carbinol extracts of *C. sativum* and *P. crispum* leaves were added to the medium and the incubation was repeated, followed by the addition of 10% 3-(4, 5-dimethylthiazolyl-2)-2, 5-diphenyltetrazolium bromide (MTT) reagent and the incubation was extended for 3 hours. The cells were then absorbed at 570 nm and 630 nm to depict the IC_50_ value. Following the MTT assay (cytotoxicity test), the cells were tested for the iron content present in them, and then the iron uptake by the cells was analyzed after treating the cells with the carbinol extracts of *C. sativum* and *P. crispum* by using the inductively coupled plasma mass spectrometry (ICPMS).

## 3. Results

### 3.1. Chlorophyll Estimation

The chlorophyll estimation of *C. sativum* and *P. crispum* leaves yielded the tabulated results when absorbed at 645 nm and 663 nm (Table 2). The amount of chlorophyll present in *C. sativum* and *P. crispum* was observed to be 1.07 mg/g and 1.82 mg/g, respectively.

### 3.2. Iron Estimation

The estimation of iron in both fresh and dried leaves of *C. sativum* and *P. crispum* gave the tabulated results (Table 3) when absorbed at 540 nm, and the calculation used for iron estimation is (observed value ÷ *n*) *x* (volume ÷ 1000) mg/ml, whereas “n” represents the volume of sample added for the analysis; in the current experiment, *n* = 3 ml. The iron content was found to be higher in both the plant leaves when processed with 30% sulfuric acid with phosphate buffer saline solution. The iron content observed in the fresh leaves was 34% higher than the iron content seen in dried *C. sativum* leaves in phosphate buffer saline, whereas fresh leaves of *P. crispum* showed a 43% higher yield. In the case of 30% sulfuric acid as a solvent, the yield of fresh leaves of *C. sativum* was 38% higher and the yield of *P. crispum* was 44% higher than the dried leaves of the respective plants. On comparing *C. sativum* and *P. crispum,* the yield of *C. sativum* was 55% higher than the iron content of *P. crispum.*

### 3.3. Molecular Docking

Based on the GC-MS analysis that was performed preliminarily, the phytochemicals obtained from *C. sativum* and *P. crispum* by using three different solvents (carbinol, petroleum ether, and water) yielded about 1761 (901 + 860) identified compounds and 37 (20 + 17) unknown compounds, respectively. Among the three solvents, carbinol was found to yield more compounds than petroleum ether and water. Carbinol extracted about 309 (304 identified + 5 unknown) compounds from *C. sativum* and 327 (325 identified + 2 unknown) compounds from *P. crispum* leaves, whereas 300 and 246 compounds were extracted using petroleum ether from *C. sativum* and *P. crispum,* respectively. About 297 and 289 compounds were extracted from *C. sativum* and *P. crispum,* respectively using water as the solvent (results obtained from preliminary work, the data has not shown). Hence, our further analysis used compounds from carbinol extracts of both *C. sativum* and *P. crispum* leaves.

Following the compound identification, based on the virtual screening, only 42 compounds were selected for molecular docking based on their pharmacokinetic and pharmacodynamic properties (Table 4). Transferrin, an iron receptor, was selected as the target, and the binding affinity was observed. The cyclopenta[c]furo[3′,2′:4,5] furo[2,3-h] [1] benzopyran-11(1h)-one, 2, 3, 6a, 9a-tetrahydro-1,3-dihydroxy-4-methoxy and 2,3-dibenzoyltartaric acid- (2R,3 R)- are the top two compounds with higher binding affinity when compared with the control drug. 2,3-Dibenzoyltartaric acid- (2R,3 R)- showed hydrogen bonds with four different amino acids: lysine, phenylalanine, glutamine, aspartic acid, and cyclopenta[c]furo[3′,2′:4,5] furo[2,3-h] [1]benzopyran-11(1h)-one,2,3,6a,9a-tetrahydro-1,3-dihydroxy-4-methoxy showed two hydrogen bonds with histidine alone, whereas the control drug, folic acid, showed four hydrogen bonds with three different amino acids, two bonds with aspartic acid, and one each with lysine and leucine (Figures 1(a) and 1(c)) of the transferrin receptor.

### 3.4. *In Vitro* Analysis

The carbinol extracts of *C. sativum* and *P. crispum* leaves were nontoxic to the Caco2 cells.  Table 5 shows the test concentration and viability rate of Caco2 cells. The cells did not show any decline in viability and subsequent cell growth has also been observed, indicating that *C. sativum* and *P. crispum* extracts enhance cell proliferation and viability.Figures 2 and 3 show the cytotoxicity tests of extracts on Caco2 cells. Followed by a cytotoxicity test, the *C. sativum* and *P. crispum* extracts showed 0.67 mg/L and 0.91 mg/L of iron concentration in their carbinol extracts, respectively, when analyzed using ICPMS. After the quantification, the iron uptake of the cells was recorded and tabulated (Table 6).

The Caco2 cells treated with iron alone failed to absorb the iron, whereas the cells treated with the extracts showed excellent iron absorption. 48.51% of the total iron added was absorbed by the cells treated with *C. sativum* extracts, and 8.24% of the iron was absorbed by the *P. crispum* extracts. The apparent permeability of the cells treated with *C. sativum* extracts was moderate (1.18 × 10^6^ cm/s) and *P. crispum* extracts showed a lower permeability rate (2.01 × 10^7^ cm/s), whereas the untreated cells did not show any permeability across the membrane (0 cm/s).

## 4. Discussion

Chlorophyll is the pigment present in plant parts that has been proved to have medicinal properties. The chlorophyll derivatives influence the metabolism of lipids in a positive manner, which can be further used in the management of obesity [13]. *C. sativum* leaves have been shown to have the highest concentrations of about 14 µg/mL and the lowest of about 9.5 µg/mL of chlorophyll [14]. About 0.42 mg/g of iron has been estimated in the leaves of *C. sativum,* whereas their seeds were composed of 0.16 mg/g of iron [15]. The *C. sativum* leaves were also found to be rich in antioxidants [16]. A chlorophyll concentration of around 16.57 ± 3.2 mg/g to 10.97 ± 2.6 mg/g has been estimated in the commercially bought *C. sativum* leaves [17]. About 2.2 mg/g of chlorophyll has been quantified from the leaves of coriander [18]. The current research on the estimation of chlorophyll in the leaves of *C. sativum* has yielded 1.07 mg/g, which is considered significant. The *C. sativum* leaves exhibited 0.835 mg/g of chlorophyll, whereas *P. crispum* leaves showed an estimate of 1.282 mg/g in their fresh leaves [19]. The leaves of chlorophyll content were found to be 0.0263 ± 0.0019 mg/g in the leaves of *P. crispum* [20]. A study by Arnold et al. [21] has revealed that the chlorophyll concentration in the leaves of *P. crispum* is 0.632 mg/g, whereas about 0.185 mg/g to 1.8 mg/mL of chlorophyll was found in the study performed by Kuzma et al. [22] and Paulert et al. [23] in the leaves of *P. crispum*. Parsley leaves were examined for chlorophyll content in their baby greens variety and showed significantly higher values, i e., 18.36 mg/g [24]. The parsley leaves showed a similar quantity of chlorophyll in the current research as well.

Iron is the micronutrient that has a major role in the chlorophyll synthesis of plants [25,26]. In human beings, the role of iron is significant. From the transportation of oxygen to tissues to storage and energy employment, iron plays an irreplaceable role in the physiological functions of the human body [27]. Iron is the major component of the hemoglobin molecule, a pigment in red blood cells that is involved in the transportation of oxygen throughout the body [28]. On examining the presence of iron, the *C. sativum* showed 0.42 mg/g in the leaves and 0.16 mg/g in the seeds [28]. Around 1.06 mg/g of iron has been estimated in the leaves of *C. sativum* in the study performed by Vanisha and Monika [29]. The leaves of *P. crispum* have been suggested to contain 6.2 mg/100g iron [30]. The iron content was also notably higher in fresh as well as dried leaves, and also in the extracts prepared by using the soxhlet extraction method, indicating the leaves of *C. sativum* and *P. crispum* are significant iron sources. On the other hand, the extracts of coriander leaves showed an effective chelating nature with iron [31], indicating the iron metabolism can be influenced by coriander leaves, whereas parsley leaves are proved to have components involved in the treatment of anxiety and depression [32]. The nanoparticles produced from the parsley leaves may be used effectively against iron deficiency, anemia condition, in rats [33]. A study by Lakshmana Prabhu et al. [34] has reported that phytochemicals such as 3,4′,5,7-tetrahydroxyflavone and quercetin have a good binding affinity when analyzed for the antiasthma properties [34]. The extracts of seeds of *C. sativum* have been examined for their anti-cancer properties *via* docking of phytochemicals, and the rutin molecule has been found to have the highest binding affinity [35]. In the present study, cyclopenta[c]furo[3′,2':4,5] furo[2,3-h] [1]benzopyran-11(1h)-one,2,3,6a,9a-tetrahydro-1,3-dihydroxy-4-methoxy and (2R,3 R)-2,3-dibenzoyltartaric acid have shown an excellent binding affinity with the transferrin receptor, suggesting the positive influence in the enhancement of iron absorption.

Caco2 cell lines have been observed to be a better way to estimate iron absorption in human cells. The bioavailability, as well as the uptake of iron by Caco2 cells, has shown a considerable outcome [36]. In addition, iron uptake by the human epithelial cells can be correlated more efficiently by using *in vitro* studies, which involve the Caco2 cell lines [36,37]. The iron uptake by Caco2 cells in the current research has also shown noteworthy results that strongly suggest the utilization of *C. sativum* and *P. crispum* leaves for the enhancement of iron absorption in human beings.

## 5. Conclusion

The chlorophyll content of *C. sativum* and *P. crispum* leaves were sufficiently significant in their concentration, suggesting the rich chlorophyll nature of these two plants. The iron concentration of these two plants was considered suggestive and higher. The number of phytoconstituents in the leaf extracts of *C. sativum* and *P. crispum* has been observed to be considerably higher in all the three solvents analyzed. Among the identified compounds, the two compounds, cyclopenta[c]furo[3′,2':4,5] furo[2,3-h] [1]benzopyran-11(1h)-one,2,3,6a,9a-tetrahydro-1,3-dihydroxy-4-methoxy and (2R,3 R)-2,3-dibenzoyltartaric acid have shown a better binding affinity with the iron-binding receptor when compared with the control drug. The *in vitro* studies yielded very suggestive results on enhancing the iron absorption efficiently in the human intestinal cells by these two plants. The iron deficiency can be effectively treated by using these two plants as the *in vitro* studies have suggested an excellent iron absorption in cells treated with plant extracts.

## Figures and Tables

**Figure 1:** Docking of compound (a) butanedioic acid, 2,3-Bis(Benzoyloxy)-, (2r,3r) (b) Cyclopenta (c) Furo[3′,2':4,5]Furo[2,3-H][1]Benzopyran-11(1h)-One,2,3,6a,9a-Tetrahydro-,3-Dihydroxy-4-Methoxy, and (d): Control drug: diclofenac with transferrin receptor.

**Figure 2:** Cytotoxicity analysis on Caco2 Cells with *C. sativum* extracts with different concentrations (a) Untreated (b) 62 5 µg/ml (c) 125 µg/ml (d) 250 µg/ml € 500 µg/ml (f) 1000 µg/ml] (Both the figures 2(a) and 3(a) are the same images of the untreated cells).

**Figure 3:** Cytotoxicity analysis on Caco2 Cells with *P. crispum* with different concentrations. (a) Untreated; (b) 62 5 µg/ml; (c) 125 µg/ml; (d) 250 µg/ml; (e) 500 µg/ml; (f) 1000 µg/ml. Both Figures 2(a) and 3(a) are the same images of the untreated cells.

**Table 1:** Scientific classification of coriander and parsley.

Classification	Coriander	Parsley
Super kingdom	Eukaryota	Eukaryota
Kingdom	Viridiplantae	Viridiplantae
Phylum	Streptophyta	Streptophyta
Subphylum	Streptophytina	Streptophytina
Class	Magnoliopsida	Magnoliopsida
Order	Apiales	Apiales
Suborder	Apiineae	Apiineae
Family	Apiaceae	Apiaceae
Subfamily	Apioideae	Apioideae
Tribe	Coriandreae	Apieae
Genus	*Coriandrum*	*Petroselinum*
Species	*Sativum*	*Crispum*

**Table 2:** Chlorophyll estimation of *C. sativum* and *P. crispum* leaves.

Sample	Absorbance at 645 nm		Absorbance at 663 nm	
*C. sativum*	0.38	**x̄** = **0.38**	0.82	**x̄** = **0.82**
	0.37		0.81	
	0.39		0.83	

*P. crispum*	0.43	**x̄** = **0.43**	0.85	**x̄** = **0.85**
	0.44		0.84	
	0.42		0.86	

Footnotes: x̄ - average				

The bold numbers has been defined in the footnotes as “average.”

**Table 3:** Iron estimation in *C. sativum* and *P. crispum* leaves.

Sample	Optical density values at 540 nm	Iron	
Estimated (mg/ml)			
Blank	0.00	0	
Standard 01 (10 *μ*g/ml standard)	0.08	0.01	
Standard 02 (20 *μ*g/ml standard)	0.16	0.02	
Standard 03 (30 *μ*g/ml standard)	0.25	0.03	
Standard 04 (40 *μ*g/ml standard)	0.31	0.04	
Standard 05 (50 *μ*g/ml standard)	0.35	0.05	
*C. sativum—*fresh (solvent: phosphate buffer saline)	0.21	0.86	**0.89**
	0.23	0.93	
	0.22	0.90	
*C. sativum—*dried (solvent: phosphate buffer saline)	0.12	0.50	**0.55**
	0.15	0.63	
	0.13	0.53	
*P. crispum*—fresh (solvent: phosphate buffer saline)	0.10	0.43	**0.44**
	0.11	0.46	
	0.10	0.43	
*P. crispum—*dried (solvent: phosphate buffer saline)	0.2	0.01	**0.01**
	0.2	0.01	
	0.3	0.02	
*C. sativum—*fresh (solvent: 30% sulfuric acid)	0.26	1.06	**1.04**
	0.26	1.06	
	0.25	1.00	
*C. sativum—*dried (solvent: 30% sulfuric acid)	0.15	0.63	**0.66**
	0.18	0.76	
	0.14	0.60	
*P. crispum—*fresh (solvent: 30% sulfuric acid)	0.12	0.50	**0.46**
	0.11	0.46	
	0.10	0.43	
*P. crispum—*dried (solvent: 30% sulfuric acid)	0.04	0.02	**0.02**
	0.04	0.02	
	0.05	0.02	

The bold numbers has been defined in the footnotes as “average.”

**Table 4:** Compounds scrutinized for molecular docking.

S. no.	Name of the compound
1	Cyclopenta[C]Furo[3′,2′:4,5] furo[2,3-h][1]benzopyran-11(1h)-one, 2,3,6a,9a-tetrahydro-1,3-dihydroxy-4-methoxy-
2	Butanedioic acid, 2,3-Bis (benzoyloxy)-, (2r,3r)
3	Benzyl beta-D-glucoside
4	1-Beta-D-Ribofuranosylimidazo[1,2 B] pyrazole-7-carbonitrile
5	(4e)-6,7-Dihydro-2,1,3-benzoxadiazol-4(5h)-one oxime
6	1,2-O-(1-Methylethylidene) hexofuranose
7	5,7-Dimethylpyrazolo[1,5-A] pyrimidin-2(1h)-one
8	4-Hydroxy-3-pentyl-cyclohexanone
9	2,4-Dihydroxy-2,5-dimethyl-3(2h)-Furan-3-one
10	2-Undecenoic acid
11	Ethyl 1-thio-Alpha-L-arabinofuranoside
12	3,5-Dodecadiyne, 2-methyl-
13	1h-Pyrazole-5-carboxamide, N-(2-hydroxyethyl)-
14	Methyl 1-methyl-3-oxocyclopentanecarboxylate
15	Butane, 2-(2,2-dichloro-1,3-dimethylcyclopropyl)-
16	Ethanimidothioic acid, 2-(dimethyl)
17	Gamma-guanidinobutyric_acid
18	Isocitronellol
19	Piracetam
20	2,3,4,5-Tetrahydroxypentanal
21	2-Amino-3-hydroxypyridine
22	Ribitol
23	2,3-Dimethylfumaric acid
24	1-Deoxy-D-arabitol
25	5-Hydroxymethylfurfural
26	Diazene, Bis(1,1-dimethylethyl)-
27	Pentanedioic acid, dimethyl ester
28	2(5h)-Furanone, 5-methyl-
29	Pyrrolidin-1-acetic acid
30	Butanedioic acid, monomethyl ester
31	2,5-Furandione
32	Dimethylamine, N-(diisopropylphosphino)methyl-
33	2-Aminoethanethiol hydrogen sulfate (ester)
34	2-Methyl-1,3,4-oxadiazole
35	N-Methoxy-N-methylacetamide
36	Ethane, 1,1-diethoxy-
37	2-Methylpyrrolidine
38	2-Propen-1-ol
39	Butane, 2-isothiocyanato-
40	2,2′-Bioxirane
41	Pyrrolidine

**Table 5:** Cytotoxicity test of *C. sativum* and *P. crispum* on Caco2 cell line.

% Viability	Test concentrations (*µ*g/ml)						
	Blank	Untreated	62.5	125	250	500	1000
*C. sativum*	-	100	110.08	111.13	110.43	114.75	108.49
*P. crispum*	-	100	108.00	116.34	117.44	125.53	105.46

**Table 6:** Iron absorption analysis.

Sample	Quantity of iron added to cells (*µ*g)	Quantified iron (mg/L)	Quantity of iron taken up by cells (*µ*g)	Iron uptake by Caco2 cells (*µ*g)
Untreated	0	0.51	**0.51**	**0**
*C. sativum* treated	1.34	1.16	**1.16**	**0.65**
*P. crispum* treated	1.82	0.66	**0.66**	**0.15**
Concentration of the extracts used: 500 *µ*g/mL				

## Data Availability

The datasets generated during and/or analyzed during the current study are available from the corresponding author on reasonable request.
